# Synthesis and Optimization of MoS_2_@Fe_3_O_4_‐ICG/Pt(IV) Nanoflowers for MR/IR/PA Bioimaging and Combined PTT/PDT/Chemotherapy Triggered by 808 nm Laser

This article has been retracted.

**DOI:** 10.1002/advs.201600540

**Published:** 2017-04-10

**Authors:** Bei Liu, Chunxia Li, Guanying Chen, Bin Liu, Xiaoran Deng, Yi Wei, Jun Xia, Bengang Xing, Ping'an Ma, Jun Lin

**Affiliations:** ^1^ State Key Laboratory of Rare Earth Resource Utilization Changchun Institute of Applied Chemistry Chinese Academy of Sciences Changchun 130022 China; ^2^ University of the Chinese Academy of Sciences Beijing 100049 China; ^3^ College of Chemistry and Life Sciences Zhejiang Normal University Jinhua 321004 China; ^4^ Institute for Lasers Photonics and Biophotonics University at Buffalo The State University of New York NY 14260 United States; ^5^ School of Physical and Mathematical Sciences Nanyang Technological University 637371 Singapore Singapore

**Keywords:** 808 nm, bioimaging, combined therapy, MoS_2_ nanoflowers, size control

## Abstract

Elaborately designed biocompatible nanoplatforms simultaneously achieving multimodal bioimaging and therapeutic functions are highly desirable for modern biomedical applications. Herein, uniform MoS_2_ nanoflowers with a broad size range of 80–180 nm have been synthesized through a facile, controllable, and scalable hydrothermal method. The strong absorbance of MoS_2_ nanoflowers at 808 nm imparts them with high efficiency and stability of photothermal conversion. Then a novel multifunctional composite of MoS_2_@Fe_3_O_4_‐ICG/Pt(IV) (labeled as Mo@Fe‐ICG/Pt) is designed by covalently grafting Fe_3_O_4_ nanoparticles with polyethylenimine (PEI) functionalized MoS_2_, and then loading indocyanine green molecules (ICG, photosensitizers) and platinum (IV) prodrugs (labeled as Pt(IV) prodrugs) on the surface of MoS_2_@Fe_3_O_4_. The resulting Mo@Fe‐ICG/Pt nanocomposites can achieve excellent magnetic resonance/infrared thermal/photoacoustic trimodal biomaging as well as remarkably enhanced antitumor efficacy of combined photothermal therapy, photodynamic therapy, and chemotherapy triggered by a single 808 nm NIR laser, thus leading to an ideal nanoplatform for cancer diagnosis and treatment in future.

## 1 Introduction

Chemotherapy, photothermal therapy (PTT), and photodynamic therapy (PDT) are three main types of cancer treatment methods, which have achieved great success in extending the lives of cancer patients.^1^, ^2^, ^3^, ^4^, ^5^, ^6^, ^7^ However, the monotherapy, though maximally optimized, generally cannot eradicate the malignant tumors completely owning to the serious metastasis of cancer and the development of drug resistance.^8^, ^9^, ^10^ Recently, many researches on using nanomaterials for therapeutic applications have shifted away from monotherapy toward the combined PTT/PDT/chemotherapy and strongly confirmed the unique advantages of the combined cancer therapy approach, such as the super‐additive anticancer effect that can greatly enhance the oncolytic efficacy, a much lower toxic side effect by reducing the use dosage of drugs, and the effective suppression of the multidrug resistance.^11^, ^12^, ^13^, ^14^ To construct this kind of combined therapy systems, well‐designed nanoscale structures with multiple integrated functionalities (including PTT agents, photosensitizers, and drugs) are required.^15^, ^16^ For example, our research group previously synthesized a kind of hollow gold nanospheres (HAuNs) coated with temperature‐sensitive poly(oligo(ethylene oxide) methacrylate‐co‐2‐(2‐methoxyethoxy)ethyl methacrylate (p(OEGMA‐*co* ‐MEMA)) for loading doxorubicin (DOX) drugs and Chlorin e6 (Ce6) photosensitizers.^16^ The as‐obtained HAuNs‐p(OEGMA‐*co*‐MEMA)‐Ce6‐DOX nanocomposites exhibited a greater chemo/PTT/PDT combined therapeutic benefit than any monotherapy alone under the 650 nm laser stimulation, well demonstrating the great advantages of multimodal combined therapeutic effects for cancer therapy.

Recently, molybdenum disulfide (MoS_2_) nanomaterials have been widely reported as promising photothermal agents benefiting from their low cost, good biocompatibility, and high NIR absorbance.^17^, ^18^, ^19^, ^20^, ^21^, ^22^ Chou et al.^22^ even demonstrated that the 2D layered MoS_2_ sheets have higher photothermal conversion ability than the commonly used graphene oxides (GOs) or gold nanoparticles (AuNPs). Based on this, some researchers focused on the synthesis of various kinds of MoS_2_‐based nanostructures for effective cancer therapy.^23^, ^24^, ^25^, ^26^ For example, Liu et al.^23^ developed LA‐PEG (lipoic acid modified polyethylene glycol) functionalized MoS_2_ nanosheets as multifunctional drug carriers for PTT/chemo‐combined therapy. Kim et al.^24^ also successfully modified polyethylenimine (PEI) and PEG onto MoS_2_ to form a kind of NIR and redox double‐stimuli controlled gene delivery. Though impressive, up to now, most of the previous reports focused on the 2D single layer nanosheets of MoS_2_, which have complex and uncontrollable synthesis processes.^18^, ^27^ Moreover, the quality of the reported MoS_2_ nanomaterials concerning their morphology, particle size distribution, surface modification, and anticancer therapeutic functions was by far not satisfying.^28^, ^29^ Therefore, it is still of great interest to provide the missing link between the general synthesis of high‐quality MoS_2_‐based nanoplatforms and their multiple promising theranostic applications.

Herein, nanoflower‐like MoS_2_ structures (labeled as MoS_2_ nanoflowers) with a broad size range from 80 to 180 nm were successfully synthesized via a facile one‐step hydrothermal method. Based on the as‐synthesized MoS_2_ nanoflowers (80 nm), a new kind of multifunctional MoS_2_@Fe_3_O_4_‐ICG/Pt(IV) (labeled as Mo@Fe‐ICG/Pt) nanocomposites is successfully fabricated by covalently grafting Fe_3_O_4_ nanoparticles with PEI functionalized MoS_2_, and then loading indocyanine green (ICG) molecules and platinum (IV) prodrugs {c,c,t‐Pt(NH_3_)_2_Cl_2_(OOCCH_2_CH_2_COOH)_2_} on the surface of MoS_2_@Fe_3_O_4_. Note that for effective anticancer treatment, Pt(IV) prodrugs can offer considerable advantage compared with the cisplatin {cis‐dichlorodiammineplatinum (II), Pt(II)} owning to their low potency that can result in fewer side effects to normal tissues. Once incubated into the intracellular environment, these Pt(IV) prodrugs can be easily reduced by physiological reductants, such as ascorbic acid and glutathione, into their cytotoxic Pt(II) form and then released from the nanocomposites.^30^, ^31^ The detailed synthetic process of Mo@Fe‐ICG/Pt nanostructure is summarized in **Figure** **1**a. Compared with the other MoS_2_‐based theranostics, this work shows the following three main advantages: (i) Various sizes of high‐quality MoS_2_ nanoflowers with extraordinary surface‐area‐to‐mass ratio can be successfully synthesized, which endow them with highly efficient loading of therapeutic molecules, such as the Fe_3_O_4_ tiny nanoparticles, ICG molecules, and Pt(IV) prodrugs; (ii) The coverage densities of the therapeutic molecules can be easily controlled by manipulating the corresponding feed ratio; and (iii) The as‐obtained MoS_2_‐based theranostic platforms exhibit fine dispersibility and favorable functionality for multimodal magnetic resonance (MR)/infrared thermal (IR)/PA bioimaging, and effective PTT/PDT/Chemo‐combined therapy, which is demonstrated by not only in vitro cell culture tests but also in vivo cancer treatment achieved upon either intratumor or intravenous administration.

**Figure 1:** a) A scheme showing the preparation process of Mo@Fe‐ICG/Pt nanocomposites. b) SEM image of MoS_2_ nanoflowers. TEM images of c) MoS_2_, d) MoS_2_‐PEI, and e) MoS_2_@Fe_3_O_4_. f) The XRD of MoS_2_ nanoflowers. g) The UV–vis–NIR absorption spectra of Fe_3_O_4_, ICG, MoS_2_‐PEI, MoS_2_@Fe_3_O_4_, and Mo@Fe‐ICG. h) Photos of Mo@Fe‐ICG aqueous solution (0.2 × 10^−3^ m of Mo) before (left) and after (right) standing for 48 h.

## 2 Results and Discussion

### 2.1 Synthesis and Characterization of Mo@Fe‐ICG/Pt

In this work, nanoflower‐like MoS_2_ structures were successfully synthesized through a novel one‐pot hydrothermal method. The Scanning Electron Microscope (SEM) and Transmission Electron Microscope (TEM) images in Figure 1b,c indicate that these MoS_2_ nanoflowers are composed of numerous well‐defined nanosheets, which is helpful for the future surface modification and drug loading. The Inductively coupled plasma mass spectrometry (ICP‐MS) can approximately determine the molecular ratio of Mo and S to be 1: 2. Also, an X‐ray diffraction (XRD) result illustrates that the crystal structures of MoS_2_ nanoflowers are 2H‐MoS_2_ phase (Joint Committee of Power Diffraction Standards (JCPDS) card No. 37‐1492). The peak at 33.4°, 40.8°, and 57.8° is corresponding to (100), (103), and (110) planes, respectively. (Figure 1f) By precisely controlling the concentrations of (NH_4_)_2_MoS_4_ and N_2_H_4_•H_2_O in the reaction system, a broad size range of MoS_2_ nanoflowers with average diameters differing from 80 to 180 nm can also be successfully synthesized for the first time (Figures S1 and S2, Supporting Information). Compared with the large MoS_2_ nanoflowers, the small ones own some distinct superiorities, such as the narrow size distribution, large specific surface, good water dispersibility, and perfect photothermal properties (Figure S3, Supporting Information). Additionally, for biomedical applications, nanocrystals with small size are more preferred.^32^, ^33^ Therefore, MoS_2_ nanoflowers with the size of 80 nm were chosen for the following experiments.

PEI was used as functional ligands to provide amine functional groups on the surface of MoS_2_ nanoflowers. After the successful modification of PEI, the morphology was not significantly changed (Figure 1d), but the mean zeta potential value increased significantly from −25.4 to +27.2 mV. The content of PEI was estimated to be 27.8 wt% by thermogravimetry analysis (Figure S4, Supporting Information). Then the tiny Fe_3_O_4_ nanoparticles (≈6 nm) were covalently grafted onto the surface of MoS_2_‐PEI (Figure 1e). Note that the amount of Fe_3_O_4_ nanoparticles in MoS_2_@Fe_3_O_4_ nanocomposites can be controlled by changing the addition amount of Fe_3_O_4_ (Figure S5, Supporting Information). In order to get enhanced magnetic performance while retain the monodispersed morphology, the amount of Fe_3_O_4_ nanoparticles in Figure S5c (Supporting Information) was chosen to be attached onto MoS_2_ nanoflowers. The corresponding high‐resolution TEM (HRTEM) image in Figure S6 (Supporting Information) clearly shows the lattice fringes of Fe_3_O_4_ with interplanar spacing of 0.253 and 0.296 nm. In addition, the high angle annular dark field scanning transmission electron microscopy and elemental mapping images of MoS_2_@Fe_3_O_4_ nanocomposites (Figure S7, Supporting Information) illustrate that Mo and S elements are distributed in the core, and the N, Fe, and O elements are well distributed on the surface of MoS_2_ nanoflowers due to the successful conjugation of PEI and Fe_3_O_4_.

Owning to the high surface area and layer‐upon‐layer structure of MoS_2_@Fe_3_O_4_, indocyanine green molecules (ICG, photosensitizers) and platinum (IV) prodrugs (Pt, chemical drugs) can be successfully grafted onto the MoS_2_@Fe_3_O_4_ step by step via strong electrostatic attraction or carbodiimide cross‐linking reaction. Both the Fourier transform infrared spectroscopy (Figure S8, Supporting Information) and UV–vis–NIR absorption analysis (Figure 1g) can confirm the successful loading of ICG owning to the existence of ICG characteristic peaks. Note that the ICG molecules are apt to self‐aggregate to form dimers or oligomers during MoS_2_@Fe_3_O_4_‐ICG (labeled as Mo@Fe‐ICG) sample preparation, resulting in a remarkable broadening and redshift in the absorption spectra.^34^, ^35^, ^36^ Additionally, the actual loading of platinum content in the nanocomposites is calculated to be 5.1 wt% by ICP‐MS. These platinum (IV) prodrugs can be reduced to cisplatin in the intracellular environment in order to exhibit anticancer activities. The dispersive property of MoS_2_@Fe_3_O_4_‐ICG/Pt(IV) (labeled as Mo@Fe‐ICG/Pt) nanocomposites was also tested. As illustrated in Figure 1h, the nanocomposites keep good dispersion after 48 h standing, thus showing a great potential to be further applied for in vitro/in vivo cancer treatments.

### 2.2 The Photothermal Property of Mo@Fe‐ICG

The UV–vis–NIR absorption spectra of the aqueous dispersions containing various concentrations of Mo@Fe‐ICG were examined in detail. As illustrated in **Figure** **2**a, the spectrum of Mo@Fe‐ICG exhibits a broad absorption in the NIR region ranging from 700 to 850 nm. With the increase of Mo concentrations from 0.0125 × 10^−3^ to 0.2 × 10^−3^ m, the UV–vis–NIR absorption intensity of Mo@Fe‐ICG increases as well. Such strong NIR absorption of Mo@Fe‐ICG motivated us to study their 808 nm induced photothermal properties. We first compared the photothermal effects of MoS_2_ and Mo@Fe‐ICG nanocomposites under the 808 nm irradiation with a power density of 0.65 W cm^−2^. As illustrated in Figure S9 (Supporting Information), the Mo@Fe‐ICG nanocomposites exhibit improved photothermal efficiency, which mainly owns to the assistant photothermal effect of ICG molecules.^37^, ^38^

**Figure 2:** a) The UV–vis–NIR absorption spectra of different concentrations of Mo@Fe‐ICG. b) Temperature variation curves of Mo@Fe‐ICG solutions with different concentrations of Mo under 808 nm (0.65 W cm^−2^). c) Temperature variation curve of Mo@Fe‐ICG (0.8 × 10^−3^ m) under 808 nm (0.65 W cm^−2^). The laser was turned off after irradiation for 8 min. d) Plot of cooling time versus negative natural logarithm of the temperature driving force. The time constant is calculated to be τ_s_ = 201 s.

The temperature variation curves of Mo@Fe‐ICG with different concentrations of Mo (0, 0.1 × 10^−3^, 0.2 × 10^−3^, 0.4 × 10^−3^, and 0.8 × 10^−3^ m) were also conducted under the 808 nm irradiation (0.65 W cm^−2^). As presented in Figure 2b, the temperature of Mo@Fe‐ICG increased in a concentration‐ and irradiation duration‐ dependent manner, indicating that the Mo@Fe‐ICG nanocomposites can rapidly and efficiently convert the 808 nm laser energy into thermal energy. The in vitro IR imagings of Mo@Fe‐ICG aqueous solutions were also carried out to monitor their real‐time temperature changes during 808 nm laser irradiation (0.65 W cm^−2^). As shown in Figure S10 (Supporting Information), the temperature increase of Mo@Fe‐ICG solutions was strongly depended on their Mo concentrations and laser irradiation time. These results kept consistent with the temperature variation curves (Figure 2b), further illustrating the good photothermal conversion ability of the as‐synthesized Mo@Fe‐ICG nanocomposites.

Additionally, according to the obtained temperature curves (Figure 2c,d), the photothermal conversion efficiency of Mo@Fe‐ICG nanocomposites is calculated to be 27.7%, which is higher than that of the widely used PTT agents, such as gold nanoshells (13.0%), gold nanorods (21.0%),^39^ copper sulfide (16.3%),^40^ or carbon sphere samples (22.2%).^41^ The photothermal stability of Mo@Fe‐ICG nanocomposites was investigated by exerting five rounds of repeated laser irradiation (808 nm, 0.65 W cm^−2^) on the Mo@Fe‐ICG aqueous solutions. As shown in Figure S11 (Supporting Information), the temperature of Mo@Fe‐ICG solutions could climb to a certain level without obvious temperature decrease. Such good irradiation‐stability of Mo@Fe‐ICG would do great benefit for the future in vitro/in vivo PTT bioapplications.

### 2.3 The Photodynamic Property of Mo@Fe‐ICG

In order to evaluate the photodynamic property of Mo@Fe‐ICG, 1,4‐diphenyl‐2,3‐benzofuran (DPBF), and 2′,7′‐dichlorofluorescin diacetate (DCFH‐DA) probes were applied for the detection of reactive oxygen species (ROS) in physiological solution and cancer cells, respectively.^42^ First, the DPBF probes, whose absorption intensity at ≈417 nm decreased irreversibly when react with the generated ROS, were mixed homogeneously with MoS_2_@Fe_3_O_4_ and Mo@Fe‐ICG aqueous solutions (100 × 10^−6^ m of Mo), and then irradiated under 808 nm laser with a power density of 0.65 W cm^−2^. As shown in **Figure** **3**a,b and Figure S12 (Supporting Information), the absorption intensity at 417 nm kept constant when incubated with MoS_2_@Fe_3_O_4_, indicating a lack of ROS generation. However, when treated with Mo@Fe‐ICG, an obvious decrease of DPBF absorption at 417 nm happened, evidencing that the ROS production was contributed to the presence of ICG molecules.

**Figure 3:** a) Absorption spectra of DPBF solution incubated with Mo@Fe‐ICG (100 × 10^−6^ m of Mo) under 808 nm irradiation for different times. b) Absorption variation trends of DPBF solutions incubated with MoS_2_@Fe_3_O_4_ and Mo@Fe‐ICG (100 × 10^−6^ m of Mo) respectively as a functional of 808 nm radiation time. Intracellular ROS detection treated with c) Control, d) MoS_2_@Fe_3_O_4_, and e) Mo@Fe‐ICG (100 × 10^−6^ m of Mo) after the 808 nm laser irradiation (1.0 W cm^−2^, 5 min).

The DCFH‐DA probes, which can be oxidized by the generated ROS into a kind of green fluorescent compound of DCF, can be applied to test the generation of ROS in Hela cells. After the incubation of MoS_2_@Fe_3_O_4_ or Mo@Fe‐ICG (100 × 10^−6^ m of Mo) for 4 h, 808 nm NIR irradiation (1.0 W cm^−2^, 5 min) was applied. Then the generated green fluorescence of DCF can be evaluated by an inverted fluorescence microscope. As shown in Figure 3c, compared with the control or MoS_2_@Fe_3_O_4_ group, a much stronger green fluorescence can be seen in the Mo@Fe‐ICG group, suggesting that Mo@Fe‐ICG nanocomposites can induce more ROS generation in Hela cells. These investigations highlight the good application prospect of Mo@Fe‐ICG as a potential 808 nm induced photodynamic agent.

Except the good photothermal and photodynamic properties, the aqueous stability or laser irradiation stability of Mo@Fe‐ICG nanocomposites also plays an important role for anticancer bioapplications. Herein, first we examined the ICG binding stability of Mo@Fe‐ICG nanocomposites. After the 48 h mild shaking of Mo@Fe‐ICG aqueous solution, the absorption spectrum of supernatant after high‐speed centrifugation showed that the released ICG amount was very limited, thus demonstrating the good ICG binding stability of Mo@Fe‐ICG nanocomposites. Then the laser irradiation stability of Mo@Fe‐ICG nanocomposites was assessed. In detail, the absorption spectra of ICG (13 × 10^−6^ m), MoS_2_@Fe_3_O_4_ (400 × 10^−6^ m of Mo), and Mo@Fe‐ICG (400 × 10^−6^ m of Mo) aqueous solutions irradiated under 808 nm NIR laser for different times were recorded in **Figure** **4**. With the irradiation time prolonging from 0 to 8 min (808 nm, 0.65 W cm^−2^), the absorption intensity of free ICG decreased obviously, while no significant difference happened in the MoS_2_@Fe_3_O_4_ and Mo@Fe‐ICG group, suggesting that a much higher irradiation‐stability can be obtained after the successful modification of ICG onto the MoS_2_@Fe_3_O_4_.

**Figure 4:** The UV–vis–NIR absorption spectra of a) free ICG, b) MoS_2_@Fe_3_O_4_, and c) Mo@Fe‐ICG aqueous solutions irradiated with 808 nm (0.65 W cm^−2^) for different times. Insets in (a) and (c) are the photos before (left) and after (right) the irradiation. d) The absorption intensity changes (at 808 nm) of MoS_2_@Fe_3_O_4_, Pure ICG, and Mo@Fe‐ICG aqueous solutions as a function of radiation time.

### 2.4 MR/IR/PA Trimodal Bioimagings

MR bioimaging method is often preferred clinically without suffering from the limited penetration depth or spatial resolution.^43^, ^44^, ^45^ In this paper, by utilizing the high transverse relaxivity of Fe_3_O_4_,^46^, ^47^ the as‐synthesized Mo@Fe‐ICG nanocomposites can be effectively applied for *T*_2_‐weighted MR imaging. As shown in **Figure** **5**a_2_, the transverse relaxivity *r*_2_ of Mo@Fe‐ICG nanocomposites has been calculated as 71.8 × 10^−3^ m s^−1^ through the curve fitting of 1/*T*_2_ relaxation time as a function of Fe concentrations (×10^−3^ m). Also, in vitro MR ‐imagings with different concentrations of Fe were carried out, which presents an obvious Fe concentration‐dependent *T*_2_ darkening effect (Figure 5a_1_). The in vivo MR imagings of tumor‐bearing Balb/c mice with and without intratumoral injection of Mo@Fe‐ICG nanocomposites (2 × 10^−3^ m of Mo, 200 µL) were illustrated in Figure 5a_3_,a_4_, which unambiguously showed a significant *T*_2_‐darking effect after the Mo@Fe‐ICG injection.

**Figure 5:** a_1_) In vitro *T*_2_ weight MR images of Mo@Fe‐ICG at different Fe concentrations. a_2_) Relaxation rate *R*_2_ (1/*T*_2_) versus different molar Fe concentrations. *T*_2_‐weighted MR images of a tumor‐bearing Balb/c mouse: a_3_) preinjection and a_4_) after injection of Mo@Fe‐ICG (2 × 10^−3^ m of Mo, 200 µL). b) Infrared thermal images of tumor‐bearing Balb/c mice injected with saline (as control group) or Mo@Fe‐ICG solutions (2 × 10^−3^ m of Mo, 200 µL) under 808 nm laser. c) The correlations between the PA values and the corresponding concentrations of MoS_2_@Fe_3_O_4_ and Mo@Fe‐ICG. The in vivo PA imagings of the tumor‐bearing mice d) before and e) after the injection of Mo@Fe‐ICG (2 × 10^−3^ m of Mo, 200 µL).

The in vivo infrared thermal images of the tumor‐bearing Balb/c mice treated with or without Mo@Fe‐ICG nanocomposites were also carried out. As shown in Figure 5b, in the control group, the temperature changed slightly even after the 808 nm laser irradiation of 300 s (1.5 W cm^−2^). However, after the subcutaneous injection of Mo@Fe‐ICG (2 × 10^−3^ m of Mo, 200 µL), the surface temperature of the tumor region rose quickly with the irradiation time increasing. Also, as expected, the local temperature of the tumor increased much higher if a stronger irradiation power density was applied. After the 808 nm laser irradiation for 300 s at a higher power density of 1.5 W cm^−2^, the local temperature rose swiftly to 65 °C, generating a sufficient photothermal conversion effect to kill the targeted tumor cells.

As a newly emerging bioimaging method, PA imaging can generate high spatial resolution images and provide inherently background‐free detection by converting irradiation laser into ultrasound emission through thermoelastic expansion.^48^ Generally speaking, the generation of PA signals is highly dependent on the optical absorption coefficient of the nanomaterials. As illustrated in Figure 1g and Figure S9 (Supporting Information), both ICG molecules and MoS_2_ nanoflowers exhibit a broad absorption in the NIR region and show highly efficient photothermal conversion abilities. Therefore, both of them can efficiently generate the acoustic waves through using the thermoelastic mechanism. Herein, the in vitro PA signal sensitivities of MoS_2_@Fe_3_O_4_ and Mo@Fe‐ICG aqueous solutions (0.2 × 10^−3^, 0.4 × 10^−3^, 0.6 × 10^−3^, 0.8 × 10^−3^, and 1.0 × 10^−3^ m of Mo) were first conducted, and the results were presented in Figures S13 and S14 (Supporting Information). An obvious Mo concentration‐dependent brightening effect can be observed. Moreover, compared with MoS_2_@Fe_3_O_4_, the Mo@Fe‐ICG performed much stronger PA signals, which mainly owns to the assistant PA activity of ICG molecules. Figure 5c also provides the correlations between the PA intensities and corresponding Mo concentrations, which clearly shows the concentration‐depended enhancement of PA signals. The in vivo PA imagings of the tumor‐bearing mice before and after the injection of Mo@Fe‐ICG were also illustrated in Figure 5d. After the Mo@Fe‐ICG injection (2 × 10^−3^ m of Mo, 200 µL), the PA signal at the tumor site was noticeably higher than the background level read before the injection (displayed by the pseudo color). These results suggest the good potential of Mo@Fe‐ICG nanocomposites for future PA bioimaging applications.

### 2.5 In vitro Cytotoxicity of Mo@Fe‐ICG/Pt

Biocompatibility is a prerequisite for biomedical applications of nanomaterials.^49^ A standard 3‐(4,5‐dimethythiazol‐2‐yl)‐2,5‐diphenyl tetrazolium bromide (MTT) assay was employed to evaluate the potential cytotoxicity of Mo@Fe‐ICG nanocomposites to L929 fibroblast cells. As shown in **Figure** **6**a, after treated with the Mo@Fe‐ICG nanocomposites for 24 h, no significant decline of cell viability was observed at an Mo concentration as high as 400 × 10^−6^ m, demonstrating the good biocompability of Mo@Fe‐ICG as therapeutic nanoplatforms.

**Figure 6:** a) In vitro cytotoxicity of Mo@Fe‐ICG against L929 cells after 24 h incubation. b) Flow cytometry analysis of Hela cells under different 808 nm NIR irradiation power densities (b_1_: 0 W cm^−2^; b_2_: 0.5 W cm^−2^; b_3_: 1.0 W cm^−2^) after incubated with Mo@Fe‐ICG/Pt (100 × 10^−6^ m of Mo). c) In vitro cytotoxicity of MoS_2_@Fe_3_O_4_, MoS_2_@Fe_3_O_4_+NIR, Mo@Fe‐ICG, Mo@Fe‐ICG+NIR, Mo@Fe‐ICG/Pt, and Mo@Fe‐ICG/Pt+NIR against HeLa cell after 24 h incubation. The cells were either exposed to 808 nm laser (1.0 W cm^−2^) for 5 min or not. d) JC‐1 probes were used as the mitochondrial membrane potential indicator through comparing the fluorescence intensity ratio of red and green. The incubation concentration of Mo@Fe‐ICG/Pt is 100 × 10^−6^ m and the 808 nm NIR irradiation power density is 1.0 W cm^−2^.

Subsequently, the Flow cytometry experiments with annexin V‐FITC/PI (Fluorescein Isothiocyanate/Propidium Iodide) double staining were carried out to evaluate the apoptosis ratio of Hela cells after the incubation of Mo@Fe‐ICG/Pt nanocomposites under 808 nm NIR laser irradiation. As seen from Figure 6b, annexin V‐FITC/PI staining of Hela cells treated with Mo@Fe‐ICG/Pt alone (100 × 10^−6^ m) without 808 nm laser irradiation showed a large viable cell population with few staining for early apoptotic, late apoptotic, and dead cells. However, after further exposure to 808 nm NIR laser for 5 min, Hela cells showed an irradiation power density‐dependent cell apoptosis. That is, when increasing the irradiation power density from 0.5 to 1.0 W cm^−2^, the ratio of the apoptosis or necrosis cells increased dramatically from 49.8% to 77.4%. Besides, the dose‐dependent cell apoptotic effect of NIR‐triggered Mo@Fe‐ICG/Pt in HeLa cells is clearly shown in Figure S15 (Supporting Information). When the concentration increased from 0 to 200 × 10^−6^ m, the ratio of the apoptosis or necrosis cells increased dramatically from 19.9% to 86.4%. These results well substantiate that the as‐synthesized Mo@Fe‐ICG/Pt nanocomposites can effectively shift the live cells to apoptosis or necrosis cells under 808 nm NIR irradiation.

A standard MTT assay together with cell morphology observation and JC‐1 staining were also performed to quantitatively or qualitatively detect the cell viabilities. First, the cytotoxic effects of different concentrations of MoS_2_@Fe_3_O_4_, Mo@Fe‐ICG, and Mo@Fe‐ICG (12.5 × 10^−6^, 25 × 10^−6^, 50 × 10^−6^, 100 × 10^−6^, and 200 × 10^−6^ m) against HeLa cells with/without 808 nm NIR irradiation (1.0 W cm^−2^, 5 min) were carefully evaluated by the MTT assay. As shown in Figure 6c, no significant cell cytotoxicity is observed after 24 h incubation of MoS_2_@Fe_3_O_4_ and Mo@Fe‐ICG without laser irradiation, confirming a well affinity between Hela cells and the samples. Mo@Fe‐ICG/Pt also demonstrates limited cytotoxic effect on Hela cells even at the concentration of as high as 200 × 10^−6^ m. However, after the 808 nm irradiation for 5 min, MoS_2_@Fe_3_O_4_+NIR, Mo@Fe‐ICG+NIR, and Mo@Fe‐ICG/Pt+NIR groups have obvious inhibitory effects on Hela cells. Moreover, it is found that the NIR‐induced cell‐killing ability arranged from high to low is MoS_2_@Fe_3_O_4_+NIR, Mo@Fe‐ICG+NIR, and Mo@Fe‐ICG/Pt+NIR under the identical conditions. For instance, the inhibitory rate of Hela cells incubated with Mo@Fe‐ICG/Pt (100 × 10^−6^ m) under 808 nm laser radiation is calculated to be 69.7%, obviously higher than MoS_2_@Fe_3_O_4_ (42.3%) and Mo@Fe‐ICG (60.4%) groups. The best cell lethality of Mo@Fe‐ICG/Pt+NIR should be attributed to the excellent PTT/PDT combined effect of MoS_2_ and ICG, together with the controlled release of Pt(II) anticancer drugs. The above MTT results can also be proved by the fluorescence microscopy images of Hela cells (Figure S16, Supporting Information). Compared with the control group, the cells treated with Mo@Fe‐ICG/Pt+NIR are round and nonadherent, revealing the serious apoptosis of cancer cells.

It is well known that the decrease of the mitochondrial membrane potential is a landmark event of early cell apoptosis.^50^ Herein, we used the fluorescent cationic dyes of JC‐1 to evaluate the Δ*Ψ*_m_ alteration of Hela cells through detecting a switch from red to green fluorescence. When the Δ*Ψ*_m_ is high, red fluorescence from Hela cells can be seen, because JC‐1 dyes can accumulate in the mitochondrial matrix to form JC‐1 aggregates. Alternatively, the JC‐1 cannot accumulate to the mitochondrial matrix, thus resulting in a green fluorescence from the JC‐1 monomers. The red or green fluorescence can be detected by an inverted fluorescence microscope. As presented in Figure 6d, the Hela cells of the control group mainly presented red fluorescence of the JC‐1 aggregates, indicating that the mitochondrial membrane potential of cells remains high. However, after 4 h incubation of Mo@Fe‐ICG/Pt (100 × 10^−6^ m), the 808 nm NIR laser irradiation (1.0 W cm^−2^, 5 min) can obviously induce the fluorescence of Hela cells change to green. That is, the low mitochondrial membrane potential happened, which represented the cell apoptosis.

### 2.6 In vivo Antitumor Efficacy of Mo@Fe‐ICG/Pt

As a proof‐of‐concept experiment, the in vivo antitumor efficacy of 808 nm irradiated PTT/PDT/chemotherapy based on Mo@Fe‐ICG/Pt nanocomposites was assessed by using H22 tumor‐bearing Balb/c mice model with administration of both intratumor and tail‐vein injection. All animal experiments were performed in compliance with the National Regulation of China for Care and Use of Laboratory Animals. First, intratumor injection was applied on seven groups (six mice in each group) of tumor‐bearing Balb/c mice: (i) Phosphate buffer saline (PBS) only (control group), (ii) NIR, (iii) Mo@Fe‐ICG, (iv) Mo@Fe‐ICG/Pt, (v) MoS_2_@Fe_3_O_4_+NIR, (vi) Mo@Fe‐ICG+NIR, and (vii) Mo@Fe‐ICG/Pt+NIR. Note that the mice were randomly divided into seven groups in order to minimize the experimental error. Moreover, the experimental conditions of each group, such as the intratumoral injection dose (2 × 10^−3^ m of Mo), injection time, 808 nm irradiation power density (1.5 W cm^−2^, 10 min), and irradiation time (6 h after the injection) also maintain a high degree of unity to produce the most accurate in vivo data possible. During the experimental time, both the mice weights and the tumor sizes were recorded every 2 d. As shown in **Figure** **7**a, the variation tendencies of the body weights in all seven groups seem similar. As the time went on, the body weights maintain within a reasonable range (20–30 g), implying that the as‐obtained samples have negligible adverse effect for in vivo applications. However, the growth trends of the tumor volumes vary significantly from each other. As plotted in Figure 7b, compared with the control group, the tumors in the NIR and Mo@Fe‐ICG groups show similar volume growth rate, suggesting that the power density of 808 nm irradiation (1.5 W cm^−2^, 10 min) as well as the dose of Mo@Fe‐ICG nanocomposites (2 × 10^−3^ m of Mo) show no obvious tumor‐inhibition effect. The mice treated with Mo@Fe‐ICG/Pt nanocomposites had a relatively better tumor inhibitory rate at early days, but followed by a rapid growth of tumor, similarly resulting in a large relative tumor volume (*V*/*V*_0_ = 16.52, *V*_0_ and *V* are the corresponding tumor volume before and after the treatment) after 18 d. In contrast, the mice treated with MoS_2_@Fe_3_O_4_+NIR, Mo@Fe‐ICG+NIR as well as Mo@Fe‐ICG/Pt+NIR presented much lower tumor growth rates. The tumor volume for the group of Mo@Fe‐ICG/Pt+NIR is the smallest (*V*/*V*_0_ = 0.23), followed by Mo@Fe‐ICG+NIR group (*V*/*V*_0_ = 2.39) and MoS_2_@Fe_3_O_4_+NIR group (*V*/*V*_0_ = 8.24).

**Figure 7:** a) The body weights and b) the relative tumor volumes of Balb/c mice after various intratumor treatments. The mice were intratumorally injected with 2 × 10^−3^ m of nanomaterials and received 808 nm irradiation (1.5 W cm^−2^, 10 min) 6 h after the injection. c) Representative photographs of mice after different intratumoral treatments. d) The photographs and the mean tumor weights of the excised tumors after various treatments. e) Hematoxylin and eosin (H&E) staining of tumor slices for control, NIR, Mo@Fe‐ICG/Pt, and Mo@Fe‐ICG/Pt+NIR groups, respectively.

The digital photos of tumor‐bearing mice after different treatments were recorded in Figure 7c, which can visually display the growth changes of tumors over time. It is worth to note that the skin of mice at the irradiation site in the Mo@Fe‐ICG/Pt+NIR group peeled off and new skin grew, further confirming that Mo@Fe‐ICG/Pt nanocomposites can lead to a good tumor‐inhibition effect. At day 18, all of mice were sacrificed and tumors were stripped. As presented in Figure 7d, both the photographs and the average tumor weights display that the tumor of Mo@Fe‐ICG/Pt+NIR group is the smallest. The H&E staining images of the representative tumor slices from different treatment groups (Figure 7e) also illustrated that most of the tumor cells were killed in the Mo@Fe‐ICG/Pt+NIR group. These results all revealed that the combined PTT/PDT/chemotherapies based on Mo@Fe‐ICG/Pt nanocomposites can achieve enhanced anticancer therapy efficiency.

Encouraged by the good therapeutic efficacy discussed above, we further assessed the in vivo antitumor efficacy of Mo@Fe‐ICG/Pt by tail‐vein injection. 24 tumor‐bearing mice were randomly divided into four groups (*n* = 6) and treated with (i) NIR‐2 only (2.5 W cm^−2^, 10 min), (ii) Mo@Fe‐ICG/Pt (2 × 10^−3^ m of Mo), (iii) Mo@Fe‐ICG/Pt+NIR‐1 (1.5 W cm^−2^, 10 min), and (iv) Mo@Fe‐ICG/Pt+NIR‐2 (2.5 W cm^−2^, 10 min), respectively. Note that two laser power densities of 1.5 and 2.5 W cm^−2^ were tested in this experiment in order to determine a better power density for achieving substantial in vivo treatment efficacy. For each mouse, the NIR irradiation was applied 12 h after the intravenous injection. The body weights and tumor size were also monitored every other day. As presented in **Figure** **8**a, the body weights of all tail‐vein injected mice show a stable increase, indicating the negligible adverse influence of nanomaterials to the mice. Additionally, the variation curves of tumor volumes within given duration are plotted in Figure 8b. After 18 d feeding, the relative tumor volumes (*V*/*V*_0_) of NIR‐2, Mo@Fe‐ICG/Pt, Mo@Fe‐ICG/Pt+NIR‐1, and Mo@Fe‐ICG/Pt+NIR‐2 were 16.9, 14.25, 8.68, and 0.06, respectively. It was found that the relative‐low power density of NIR‐1 (1.5 W cm^−2^) can only partially damage the tumor, which is insufficient for tumor ablation. This is mainly due to the insufficient accessibility and accumulation of MoS_2_@Fe_3_O_4_‐ICG/Pt nanocomposites into the tumor site after the intravenous injection. When properly increasing the irradiation power density to NIR‐2 (2.5 W cm^−2^), the tumor treated with Mo@Fe‐ICG/Pt shrank significantly, just leaving a black scar on the tumor location after 18 d (Figure 8c). The H&E staining images of the representative tumor slices (Figure 8d) also illustrated that a serious cancer cell necrosis happened in the Mo@Fe‐ICG/Pt+NIR‐2 group. These in vivo experimental results again confirm that our design of the combined PTT/PDT/chemotherapies based on Mo@Fe‐ICG/Pt nanocomposites have great potential for the future utilization as efficient antitumor agents.

**Figure 8:** a) The body weights and b) the relative tumor volumes of Balb/c mice after various tail‐vein injection treatments. c) Representative photographs of mice after different tail‐vein injection treatments. d) Hematoxylin and eosin (H&E) staining of tumor slices for NIR‐2, Mo@Fe‐ICG/Pt, Mo@Fe‐ICG/Pt+NIR‐1, and Mo@Fe‐ICG/Pt+NIR‐2 groups, respectively. The injection concentration is 2 × 10^−3^ m of Mo, and the NIR‐1 and NIR‐2 represent 808 nm laser with a power density of 1.5 and 2.5 W cm^−2^, respectively.

### 2.7 The Potential Toxicity of Mo@Fe‐ICG

Since the potential toxicity of the nanomaterials plays an important role for their future clinical applications,^51^, ^52^ some physiological parameters of Balb/c mice, such as the serum biochemistry, hematoxylin and eosin (H&E) staining of main organs, and the weight fluctuations, after the injection of Mo@Fe‐ICG nanocomposites (2 × 10^−3^ m of Mo) were carefully monitored. Note that during the entire experimental period, all the mice performed well without any observable sign of toxic effects.

The serum biochemistry test of mice was first carried out on the day 1, day 3, and day 7 after the intravenous injection of Mo@Fe‐ICG nanocomposites. As shown in **Figure** **9**a–d, various kinds of biochemical parameters have been tested, including the alanine aminotransferase and aspartate aminotransferase (ALT and AST, both are liver function signals), blood urea nitrogen and creatinine (CRE and BUN, both are kidney function indicators), and creatine kinase (CK, heart function maker). Encouragingly, the tested parameters show no significant difference between control group and Mo@Fe‐ICG group, indicating that no obvious liver, kidney, or heart damage happened after the intravenous injection of Mo@Fe‐ICG nanocomposites. Afterward, H&E staining images of the representative main organ slices, such as the heart, liver, spleen, lung, and kidney, were performed after the intratumor or tail‐vein injection of Mo@Fe‐ICG nanocomposites. As presented in Figure S17 (Supporting Information) and Figure 9e, compared with the control group, neither organ damage nor inflammatory lesion can be observed in the detected organs after the intratumor or tail‐vein injection of Mo@Fe‐ICG, proving the low in vivo toxicity of Mo@Fe‐ICG at the tested dose for future anticancer bioapplications. Moreover, the weights of healthy Balb/c mice intravenously injected with different doses of Mo@Fe‐ICG nanocomposites (0.16, 0.32, and 0.64 mg per mouse) were also monitored every 2 d and the results are recorded in Figure S18 (Supporting Information). It can be seen that the body weight fluctuations of mice after Mo@Fe‐ICG injection show no noticeable difference with the control group (with PBS injection), again demonstrating the good biosecurity of Mo@Fe‐ICG for future bioapplications.

**Figure 9:** a–d) Serum biochemistry data including alanine aminotransferase (ALT), aspartate aminotransferase (AST), blood urea nitrogen (BUN), creatinine (CRE), and creatine kinase (CK). e) H&E staining images of the representative main organ slices, such as the heart, liver, spleen, lung, and kidney after the tail‐vein injection of Mo@Fe‐ICG (2 × 10^−3^ m of Mo).

The in vivo long‐term tissue biodistribution of Mo@Fe‐ICG nanocomposites was also conducted.^53^ In detail, 24 healthy Balb/c mice were tail‐vein injected with Mo@Fe‐ICG nanocomposites and then euthanized at different time points (1, 3, 12 h, 1, 3, and 7 d). The major organs (heart, liver, spleen, lung, and kidney) of each mouse were collected and treated with HNO_3_ and H_2_O_2_ (v/v = 1:1) at 60 °C to obtain clear solutions. Finally, the Mo concentrations in the solutions were determined by ICP‐MS. As given in **Figure** **10**, at the early stage of intravenous injection, Mo@Fe‐ICG nanocomposites were taken up mainly by the liver, spleen, and lung of the Balb/c mice. As the extension of time, obvious decrease of Mo concentrations occurred in all the tested organs, illustrating that the nanocomposites could generally be excreted from the mice as time prolonging. These results can help us relieve the concerns on the toxicity of the as‐synthesized Mo@Fe‐ICG nanocomposites for in vivo bioapplications.

**Figure 10:** The in vivo biodistribution of Mo element after injecting Mo@Fe‐ICG nanocomposites (2 × 10^−3^ m of Mo) intravenously at different time points.

## 3 Conclusion

In summary, MoS_2_ nanoflowers with a broad size range differing from 80 to 180 nm were successfully synthesized via a facile one‐step hydrothermal method. The strong absorbance of MoS_2_ nanoflowers in the near‐infrared range imparts them with high efficiency and stability of photothermal conversion. Based on these MoS_2_ nanoflowers, a new kind of multifunctional MoS_2_@Fe_3_O_4_‐ICG/Pt(IV) (labeled as Mo@Fe‐ICG/Pt) nanocomposites is successfully fabricated by covalently grafting Fe_3_O_4_ nanoparticles with PEI functionalized MoS_2_, and then loading ICG molecules and platinum (IV) prodrugs on the surface of MoS_2_@Fe_3_O_4_. The photothermal/photodynamic property, MR/IR/PA trimodal bioimagings, in vitro/in vivo antitumor efficacy as well as the potential long‐term toxicity of nanocomposites have illustrated in detail. The results show that the as‐fabricated Mo@Fe‐ICG/Pt nanocomposites exhibit good MR/IR/PA trimodal imaging capacity and remarkable PDT/PTT/chemo‐combined effect, thus resulting in an ideal treatment efficacy for complete eradication of solid tumors.

## Supporting information

Supplementary
